The article "The Novel Sensor Network Structure for Classification Processing Based on the Machine Learning Method of the ACGAN" was retracted in 2020. Reasons: plagiarism; overlap with other authors' work.

# The Novel Sensor Network Structure for Classification Processing Based on the Machine Learning Method of the ACGAN

**DOI:** 10.3390/s19143145

**Published:** 2019-07-17

**Authors:** Yuantao Chen, Jiajun Tao, Jin Wang, Xi Chen, Jingbo Xie, Jie Xiong, Kai Yang

**Affiliations:** 1 School of Computer and Communication Engineering & Hunan Provincial Key Laboratory of Intelligent Processing of Big Data on Transportation, Changsha University of Science and Technology, Changsha 410114, China; 2 School of Information Science and Engineering, Fujian University of Technology, Fuzhou 350118, China; 3 Hunan Institute of Scientific and Technical Information, Changsha 410001, China; 4 Electronics & Information School, Yangtze University, Jingzhou 434023, China; 5 Technical Quality Department, Hunan ZOOMLION Heavy Industry Intelligent Technology Corporation Limited, Changsha 410005, China

**Keywords:** generative adversarial networks (GAN), auxiliary classifier generative adversarial networks (ACGAN), feature matching, image classification, CP-ACGAN

## Abstract

To address the problem of unstable training and poor accuracy in image classification algorithms based on generative adversarial networks (GAN), a novel sensor network structure for classification processing using auxiliary classifier generative adversarial networks (ACGAN) is proposed in this paper. Firstly, the real/fake discrimination of sensor samples in the network has been canceled at the output layer of the discriminative network and only the posterior probability estimation of the sample tag is outputted. Secondly, by regarding the real sensor samples as supervised data and the generative sensor samples as labeled fake data, we have reconstructed the loss function of the generator and discriminator by using the real/fake attributes of sensor samples and the cross-entropy loss function of the label. Thirdly, the pooling and caching method has been introduced into the discriminator to enable more effective extraction of the classification features. Finally, feature matching has been added to the discriminative network to ensure the diversity of the generative sensor samples. Experimental results have shown that the proposed algorithm (CP-ACGAN) achieves better classification accuracy on the MNIST dataset, CIFAR10 dataset and CIFAR100 dataset than other solutions. Moreover, when compared with the ACGAN and CNN classification algorithms, which have the same deep network structure as CP-ACGAN, the proposed method continues to achieve better classification effects and stability than other main existing sensor solutions.

## 1. Introduction

Image classification algorithms have always been a hot research topic in the field of image processing research. Krizhevsky et al. [1] proposed the AlexNet network, based on deep learning methods, which has been successfully applied to image classification in the ImageNet dataset [1]. The Top5 error rate was controlled at the 15.4% level, a full ten percentage points higher than the non-deep learning method that took second place. Moreover, ResNet [2] controlled the Top5 error rate at the 3.57% level, which exceeds the performance of human recognition. The successful application of these deep networks has caused deep convolutional neural networks (DCNNs) to gradually become one of the most important methods in the field of image classification research. DCNNs are essentially a more effective feature extraction method that takes the extracted features as the input of a classifier to achieve image classification. However, the major drawback of such networks is that they can only use artificially supplied samples; moreover, the models cannot learn the spatial distribution of samples. In addition, the distribution between samples cannot account for a deeper understanding of the sample’s internal structure, which will undoubtedly affect the model’s image classification performance.

The article "The Novel Sensor Network Structure for Classification Processing Based on the Machine Learning Method of the ACGAN" was retracted in 2020. Reasons: plagiarism; overlap with other authors' work.

The generative model is a model that can learn the potential distribution of data and generate new sensor samples. Traditional generative models include the Gaussian model (GM), Bayesian network (BN) [3], S-type reliability network (SRN) [4], Gaussian mixture model (GMM) [5], multinomial mixture model (MMM) [6], hidden Markov model (HMM) [7] and hidden Markov random field (HMRF) [8]. Goodfellow et al. [9] proposed generative adversarial networks (GAN) by summarizing the advantages and disadvantages of traditional generative networks. The main idea behind the GAN model involves training two antagonistic networks simultaneously: namely, a generative network (G) and discriminative network (D). The key aspect of training a discriminative network is that it can distinguish real sensor samples from the pseudo-samples generated by the generative network, which is defined as binary classification. Accordingly, the generative network is trained to generate sensor samples that look as real as possible, with the aim of causing the discriminative network to mistake them for real sensor samples, thereby achieving the effect of false and fake.

Subsequently, Radford et al. [10] proposed deep convolutional generative adversarial networks (DCGAN), which combine GAN with a convolutional neural network (CNN) in order to make the process of training the generative network more stable and arrive at a clearer generated image. Furthermore, Mirza et al. [11] proposed conditional generative adversarial networks (CGANs). Unlike the original GAN model, CGANs are trained by adding class labels to both the generator and discriminator, thus realizing directional image generation. Odena et al. [12] further proposed the ACGAN network. Like the CGAN model, the ACGAN model uses image label information during the training procedure; however, it only adds label information to the generator to realize directional image generation. Experimental results have shown that the ACGAN can generate samples with higher definition. The traditional GAN belonged to the unsupervised learning method category. While Kingma et al. [13], Gui et al. [14], Zhang et al. [15] and Xia et al. [16] successfully applied the GAN model to a semi-supervised learning procedure, the application of the CGAN and ACGAN brings it into supervised learning territory. Salimans et al. [17] proposed an image recognition method based on the CGAN model. The GAN has been successfully applied to supervised image classification. The traditional discriminator of the ACGAN network is the natural classifier; however, when used in image classification applications, many problems arise including unstable training, poor discriminative effects and so on [18,19,20,21,22].

The article "The Novel Sensor Network Structure for Classification Processing Based on the Machine Learning Method of the ACGAN" was retracted in 2020. Reasons: plagiarism; overlap with other authors' work.

Based on the above problems, the present paper proposes classification processing based on an auxiliary classifier generative adversarial network (CP-ACGAN). The proposed method adjusts the sensor structure of the ACGAN network in several key ways. Firstly, the real discrimination and fake discrimination of sensor samples has been canceled in the discriminator (D), and only the prediction vectors of labels in sensor samples are outputted. Secondly, the pooling and caching method of the CNN is fused with the ACGAN model. That is, the convolutional layer part of the discriminator in the ACGAN is changed into a pooling layer so that the diversity of generative networks can be effectively utilized, while the feature extraction ability of the pooling method can also be utilized to achieve a better classification effect. Thirdly, feature matching (*FM*) is also proposed to improve the diversity of the generated samples. The proposed algorithm has been proven to be an effective classification method for semi-supervised learning procedures. Experimental results have shown that the proposed algorithm (CP-ACGAN) yields a better classification performance than the ACGAN method. At the same time, when compared with a CNN with a sensor network structure, it also achieves better classification accuracy. Therefore, the CP-ACGAN image classification method proposed in the present paper represents an improved image classification algorithm. Moreover, improving both the generator and the diversity of the generative sensor samples can further improve the network classification effect.

The article "The Novel Sensor Network Structure for Classification Processing Based on the Machine Learning Method of the ACGAN" was retracted in 2020. Reasons: plagiarism; overlap with other authors' work.

The rest of this paper is organized as follows. Section 2 discusses the GAN and its deformation. In Section 3, we propose the classification processing algorithm based on the ACGAN. Section 4 mainly deals with the experimental results of the paper. Finally, Section 5 presents the conclusion and some suggested avenues for future work.

## 2. Generative Adversarial Networks and Their Deformation

### 2.1. Generative Adversarial Networks

The generation of confrontational networks is one of the generative models proposed by Goodfellow et al. [9]. The GAN model is based on the minimum and maximum problem of the two-person game. The method of confrontation training is as shown in Equation (1):

(1) $$\underset{G}{\min}\underset{D}{\max}V(G,D)=E_{x\sim p_{data}}[\log D(x)]+E_{z\sim p_{z}(z)}[\log(1-D(G(z)))]$$

The network structure of the GAN model is presented in Figure 1 above. $N_{z}$ represents noise information. $X_{real}$ is the real sample and $X_{fake}$ is the virtual sample. Real/Fake is the optional result of the output. The GAN network model consists of a generator (*G*) and discriminator (*D*); here, the generator (*G*) conducts mapping from $z\sim p_{z}(z)$ noise to generate sensor sample space $G(z;\theta_{g})$, while the discriminator $D(x;\theta_{d})$ determines whether the input x has come from real sensor samples or generated sensor samples, meaning that the discriminator essentially has two classes. In the continuous confrontation between *G* and *D*, the generation $p_{g}(x)$ of the distribution comes to approximate the real distribution of p(x), and ultimately achieves a Bayesian Nash equilibrium. At this time, the generator can match the real data distribution completely; that is, $p_{g}(x)=p(x)$, while the discriminator is $D(x)=p(x)/(p_{g}(x)+p(x))=1/2$. Thus, the distribution of generated samples is completely consistent with that of the real samples, and the purpose of generating real samples has been achieved. Both neural networks (*G* and *D*) of the GAN model make use of the traditional back-propagation principle, and the computational processing requires neither complex Markov chains nor maximum relief estimation; nor does it exhibit a complex variation in lower bounds, which greatly reduces the difficulty of network training and makes it easier to achieve convergence.

### 2.2. Deep Convolutional Generative Adversarial Networks

The generator (*G*) and discriminator (*D*) of the original GAN model are all fully based on connected neural networks. The training procedure is simple and the amount of calculations required is small; however, the images generated after training are blurred and the obtained visual effects are poor. Furthermore, a CNN has a powerful feature extraction ability and better spatial information perception ability. Radford et al. [10] first proposed the DCGAN network model. In the DCGAN model, the convolutional layer and transposed convolutional layer are used to replace the fully connected layers in the generator (*G*) and discriminator (*D*), respectively, so that the generated image has higher definition [23,24]. The DCGAN is characterized by the following changes in network structure:

(1). The pooling layer in the CNN has been canceled; strided convolutions are used in the discriminator, while fractional strided convolutions are used in the generator (*G*).
(2). In addition to the generative output layer and the discriminative input layer, another layer has been added, namely a batch norm (BN). The BN can help to reduce the excessive dependence of the network on the initial parameters, as well as prevent the initialization parameters from being subpar. It further prevents the gradient from disappearing and transfers the gradient to each layer of the network; moreover, it prevents the generator from converging to the same point, thereby improving the diversity of the generated samples. This also reduces the network oscillation and improves the stability of network training.
(3). The full connection layer has also been cancelled. In the generator (*G*), while the activation function *Tanh* is used in the final output layer, the activation function *ReLU* is used in all other layers. The leaky activation function *ReLU* is used in all layers of the discriminator.

The article "The Novel Sensor Network Structure for Classification Processing Based on the Machine Learning Method of the ACGAN" was retracted in 2020. Reasons: plagiarism; overlap with other authors' work.

### 2.3. Auxiliary Classifier Generative Adversarial Networks

The traditional generative networks were unsupervised models. The CGAN applied the generated antagonistic network concept to the supervised learning method for first time, allowing it to achieve a corresponding effect between tags and generated images. The ACGAN [16] was further improved on the basis of the CGAN through incorporation of the idea of mutual information in InfoGAN [25]. $N_{z}$ represents noise information and $L_{y}$ is the label used by the generator (*G*). $X_{real}$ is the real sample and $X_{fake}$ is the virtual sample. Real/Fake is the optional result of the output. $L_{y{}^{\prime }}$ is the output label used by the discriminator (*D*). The network structure of the ACGAN is shown in Figure 2 below.

Equations (2) and (3) are the objective functions of the ACGAN training process:

(2) $$L_{s}=E[\log p(s=\mathrm{real}|x_{data})]+E[\log p(s=\mathrm{fake})|x_{fake}]$$

(3) $$L_{c}=E[\log p(C=c|x_{data})]+E[\log p(C=c)|x_{fake}]$$

*D* is trained to maximize $L_{s}+L_{c}$, while *G* is trained to maximize $L_{s}-L_{c}$. From the network structure or from training the objective function, we can see that the loss function of the ACGAN model has incorporated the cross-entropy between the input sample label information and the label posterior probability estimation value on the basis of the GAN model [26,27].

The article "The Novel Sensor Network Structure for Classification Processing Based on the Machine Learning Method of the ACGAN" was retracted in 2020. Reasons: plagiarism; overlap with other authors' work.

## 3. Image Classification Processing Algorithm Using ACGAN

### 3.1. Applied ACGAN for Image Classification

The discriminator in the ACGAN outputs the posterior error estimate of the input tag, as well as the real and fake discrimination of the output sample. After the network training is complete, input the sample x; the discriminator can then output its corresponding probability p(y|x) for each class and select the category p(y|x), which makes k the largest and thus the label of the input sample x, so as to achieve image classification operation.

The generator structure of the ACGAN-based image classification model is presented in Figure 3 (the example dataset is MNIST). The network generator consists of four fully connected layers and five transposed convolutional layers. The structure of transposed convolutional layers one and three is the same (kernel_size is 4, stride is 2, padding is 1), while that of transposed convolutional layers two, four, and five are also the same (kernel_size is 5, stride is 1, padding is 1).

Figure 4 presents the discriminator structure diagram of the ACGAN model. The discriminator has the contrary structure to the generator, as it comprises five convolutional layers and four fully connected layers. Here, convolutional layers one, two and four have the same structure (kernel_size is 5, stride is 1, padding is 1), while convolutional layers three and five have the same structure (kernel_size is 4, stride is 2, padding is 1). The output layer of the discriminant network outputs the posterior probability estimation of the sample label; that is, the estimated value of the sample label in the testing dataset, in addition to the authenticity discrimination of the output sample. The ACGAN [16] is based on adding label constraints to improve the quality of high-resolution image generation, and it can propose a new measurement of image quality and mode collapse.

### 3.2. The CP-ACGAN Algorithm

#### 3.2.1. Feature Matching Operation

The feature matching (FM) operation is the proposed method utilized by the improved GAN to enhance training stability and generate sample diversity. Assuming that f(x) represents the discriminator output of the middle layer, the objective function of FM can be expressed by means of Equation (4):

(4) $$\min_{\theta_{g}}={\left\|E_{x\sim p_{\mathrm{data}}}[f(x)]-E_{z\sim p_{z}}[f(G(z))]\right\|}_{2}^{2}$$

The feature output of the generated sample in the discriminator matches the feature output of the real sample in the discriminator. While Salimans et al. [17] and Zhang et al. [28] indicated that minibatch discrimination [29] can produce better results under some circumstances, feature matching achieves a better classification effect under semi-supervised learning conditions. Therefore, the present paper opts to introduce feature matching into the ACGAN to further improve its image classification performance.

The article "The Novel Sensor Network Structure for Classification Processing Based on the Machine Learning Method of the ACGAN" was retracted in 2020. Reasons: plagiarism; overlap with other authors' work.

#### 3.2.2. Improved Loss Function

Some potential problems with the proposed configuration were identified, including slow training speed, unstable network and poor effect when using the ACGAN discriminant network *D* to classify images. Therefore, the original ACGAN network structure has been improved. $N_{z}$ represents noise information and $L_{y}$ is the label used by the generator (*G*) and $X_{real}$. $X_{real}$ is the real sample and $X_{fake}$ is the virtual sample. $y{}^{\prime }$ is the predicted value of the sample label. The improved network structure is presented in Figure 5.

In terms of the network structure, the improved network cancels the real and fake samples of the discriminant in the discriminator, as well as introducing feature matching in the discriminator, although the other parts remain unchanged. However, in order to ensure the effective use of the real and fake samples, the loss function of the generator and discriminator has been substantially altered. The real samples are now treated as labeled supervisory data, while the generated samples are treated as labeled fake data. The softmax classifier is then connected to the output layer of the discriminant network. The supervisory loss function of the real samples can be expressed as Equation (5):

(5) $$\begin{array}{ll} L_{\mathrm{supervised}} & =-E_{(x,y)\sim p_{\mathrm{data}}}[\log p(y|x,y<K+1)]\\ \; & =-\frac{1}{N}\log p(y|x,y<K+1)\\ \; & =-\frac{1}{N}\log\frac{\exp(\langle y,y{}^{\prime }\rangle )}{\sum_{i=1}^{K}\exp y_{i}^{\prime }}\\ \; & =-\frac{1}{N}(\langle y,y{}^{\prime }\rangle +\log(\sum_{i=1}^{K}\exp y_{i}^{\prime }))\\ \; & =CE(y,y{}^{\prime }) \end{array}$$

Here, N is the batch size of samples, 〈⋅ , ⋅〉 is the inner product, y is the sample label, and $y{}^{\prime }$ is the predictive value of the sensor label. Therefore, the loss function of the real data can be expressed as Equation (6):

(6) $$L_{\mathrm{real}}=L_{\mathrm{supervised}}$$

For data generation, the error consists of two parts: one is the probability loss value of the false sample K+1 class, and the other is the cross-entropy of the loss value between the output label $y_{\mathrm{fake}}^{\prime }$ and the input label y. Let $L_{unsupervised}$ express the probability of expected loss of fake sample classes; we can then make use of the property of the softmax function to make $y_{K+1}^{\prime }=0$ and obtain Equation (7):

(7) $$\begin{array}{ll} L_{\mathrm{unsupervised}} & =-E[\log p(y=K+1|x)]\\ \; & =-\frac{1}{N}\log p(y=K+1|x)\\ \; & =-\frac{1}{N}\log\frac{\exp y_{K+1}^{\prime }}{\sum_{i=1}^{K+1}\exp y_{i}^{\prime }}\\ \; & =\frac{1}{N}\log(1+\sum_{i=1}^{K}\exp y_{i}^{\prime }) \end{array}$$

Because the ACGAN network is being used, the input labels of the generated samples in each batch are consistent with the labels of real samples. Therefore, the cross-entropy loss value between the generated tag $y_{\mathrm{fake}}^{\prime }$ and the input tag y is $CE(y,\;y_{\mathrm{fake}}^{\prime })$. In short, the loss of generated samples can be expressed as Equation (8):

(8) $$L_{\mathrm{real}}=0.5(L_{\mathrm{unsupervised}}+CE(y,y_{\mathrm{fake}}^{\prime }))$$

Moreover, because the parameters of the generator and discriminator are updated constantly during training, the errors of the generator and discriminator need to be constructed separately. For the discriminator *D*, the error can be expressed as Equation (9):

(9) $$L_{D}=0.5(L_{\mathrm{real}}+L_{\mathrm{fake}})$$

While for the generator *G*, the error can be expressed as Equation (10):

(10) $$L_{G}=0.5(L_{\mathrm{FM}}+L_{\mathrm{unsupervised}})$$

In addition, $L_{\mathrm{FM}}={\left\|E_{x\sim p_{\mathrm{data}}}[f(x)]-E_{z\sim p_{z}}[f(G(z))]\right\|}_{2}^{2}$ represents the two-norm loss item of feature matching.

The article "The Novel Sensor Network Structure for Classification Processing Based on the Machine Learning Method of the ACGAN" was retracted in 2020. Reasons: plagiarism; overlap with other authors' work.

#### 3.2.3. The Pooling Method

Convolutional neural networks (CNNs) have achieved great success on image classification tasks, and the pooling method has played an important role in image processing. As an important step in a CNN, the pooling method can not only extract effective features, but can also reduce the dimensionality of data and prevent the overfitting phenomenon from occurring [30]. The pooling method, which is the key step in feature extraction using a CNN, has the characteristics of translation, rotation and scaling invariance [31,32,33]. Commonly used pooling methods include mean pooling, maximum pooling and random pooling.

In the application of the GAN model, in order to make the generated image more high-definition, the use of deconvolution (Deconv) rather than the pooling method in the discriminant network has caused pooling to be abandoned in the production network. However, the pooling method has played an incomparable role in solving classification problems. Therefore, if the pooling method was to be combined with a generative confrontational network, the resulting generative confrontational network with pooling method could be used to solve classification problems effectively. On the one hand, the diversity of generative samples can be used. On the other hand, the pooling method can be used to more effectively take the features.

The article "The Novel Sensor Network Structure for Classification Processing Based on the Machine Learning Method of the ACGAN" was retracted in 2020. Reasons: plagiarism; overlap with other authors' work.

Accordingly, the present paper proposes the CP-ACGAN as a means of solving image classification problems. On the basis of introducing the feature matching and reconstruction loss functions, the convolutional layer of the discriminator in the ACGAN is changed to a pooling layer. Moreover, corresponding to Figure 4, the third and fifth convolutional layers in the original discriminant network are changed to pooling layers, while the generator structure remains unchanged. Figure 6 presents a structural diagram of the CP-ACGAN discriminant network.

### 3.3. Details of the Proposed Algorithm

In order to solve the problems proposed in Section 2.2, this paper uses a logarithmic function, represented by He et al.’s [2] total variation model. In order to reduce the illumination direction of the noise and maintain the consistency of the structure, it aims to restore image structure texture decomposition using the structural component to obtain the image illumination direction information. The priority function is also modified to improve the robustness and reliability of computation. The local model is then constructed to select the best matching block in order to ensure local structural consistency and visual credibility of the image.

The structural component *u* of the image is obtained by the logarithmic total variation minimization model. *u* is the piecewise smooth part of image *f*, including the geometric structure and equal illumination information. The texture components include small size details and random noise in the image, such as those discussed by Dong et al. [34], Lim et al. [35] and Kumar et al. [36].

Assuming that the original image is *f*, the structural component is *u* and the texture component is *v*, *U* can thus be represented as BV(Ω) (bounded variation). *U* retains the sharp edge and contour information of the image, but can remove the texture and noise components. The residual v=f−u is the generalization function defined on $L^{2}(\Omega )$. The structural texture decomposition of the images can be solved by the following convex minimization problem, defined as Equation (11):

(11) $$\inf\;F(u)=\int \left(\phi \left|\nabla u\right|\right)dx+\lambda \int_{}{\left|f-u\right|}^{2}dx$$

λ is the harmonic parameter, which controls the approximate degree of the structural component *u* and the original graph. ∫ϕ(|∇u|)dx is the generalized total variation of image *u*, and ϕ(|∇u|) is the convex function of |∇u|. The Euler Lagrange equation is satisfied by the upper minimum.

(12) $$\left\{ \begin{array}{l} \frac{\partial u}{\partial t}=\nabla (\frac{\phi {}^{\prime }\left|\nabla u\right|}{\left|\nabla u\right|}\nabla u)-\lambda_{E}(u-u_{0})\\ u(x,y)|{}_{t=0}=u_{0} \end{array}\right.$$

Here, the equation for calculating the priority term is P(p)=C(p)⋅D(p). C(p) is the confidence term and D(p) denotes the data items. The equation for calculating the confidence term is as follows:

(13) $$C(p)=\frac{\sum_{q\in N_{p}\cap \Phi }C(q)}{\left|N_{p}\right|}$$

where ψ(p) has been located, the region has been expressed in $N_{p}$. The denominator $\left|N_{p}\right|$ represents the number of image pixels in the ψ(p) piece. C(q) represents the confidence of *Q*. If it is to be repaired, it is zero, while if it is the source image area, it is one. Therefore, the molecules in Equation (1) represent the number of data points that do not need to be repaired in image slice ψ(p). The meaning of one is that there are enough real data points in the image of ψ(p) to be repaired. The more real information that the image slice provides, the higher the reliability, and it should be repaired first. The equation used to calculate data item D(p) is as follows:

(14) $$D(p)=\frac{\left|{\vec{\nabla I_{p}}}^{⊥}\cdot \vec{n_{p}}\right|}{\alpha }$$

The total variation based on the logarithmic function is $\phi (s)=\frac{1}{2}s\ln(1+s)$. It is proved that the model is an anisotropic diffusion model. Diffusion has achieved excellent performance in illumination direction and gradient direction applications. The diffusion along the direction of irradiance diffuses faster than the total variation minimization model P–M (Perna–Malik) and the anisotropic diffusion model. Accordingly, this paper can adopt the structure decomposition model of image texture. In terms of numerical calculation, the iterative Gauss–Jacobi method is adopted by introducing a half pixel point; the specific method is taken from Min et al. [37].

The article "The Novel Sensor Network Structure for Classification Processing Based on the Machine Learning Method of the ACGAN" was retracted in 2020. Reasons: plagiarism; overlap with other authors' work.

After getting the structural image of the restored image, we can calculate the priority on the structural image *u* directly. In order to overcome the influence of product effect, we modify the priority calculation rule by means of Equation (15):

(15) P(p)=ξC(p)+(1−ξ)D(p)

Here, the weight value ξ is controlled by the emphasis of C(p) and D(p), where ξ=0.5 is selected. We can thus calculate confidence in the structural image and remove the interference of some local fine-texture noise while avoiding high-priority points; when the confidence of data items is very small, the calculation of priority items is more credible than in other cases.

As described in Section 2.1, the selection of an optimal matching block with reference only to the minimum of the sum of square differences (SSD) criterion will bring about some error matching and accumulation errors. Thus, we here propose the optimal matching optimization model. The idea of the model is based on the premise of image classification. The texture structure of natural images has local continuity; the closer the distance, the more consistent the texture should be, and the smaller the total local variation of the image. Therefore, a 0-1 optimal model is proposed in this paper. The local window of the *p* point to be repaired is taken as $W_{p}$ to calculate the local total variation. The local total variation is related to the image slice ψ(p) of the repaired *p* point. According to the principle of SSD, we calculate the minimum *k* SSD image fragment as $\psi_{q_{1}},\psi_{q_{2}},\cdots ,\psi_{q_{k}}$. If $\psi (p)=\psi_{q_{i}}$ is recorded, the image of effective pixels in $W_{p}$ is totally changed into ${\mathrm{TV}}_{\mathrm{Local}}(p,i)=\int_{i\in [1,k]}\left|\nabla u_{i}\right|dx$.

Objective Function: ${\min:\mathrm{TV}}_{\mathrm{Local}}(p,i)=\int_{i\in [1,k]}\left|\nabla u_{i}\right|dx,x\in W_{p}\cap \Phi$

Decision Variables: $c_{i},i=1,2,\cdots ,k$

(16) $$s.t.\left\{ \begin{array}{l} \psi (p)=\sum_{i=1}^{k}c_{i}\psi_{q_{i}},\\ \sum_{i=1}^{k}c_{i}=1,\\ c_{i}=\{0,1\},i=1,2,\cdots ,k. \end{array}\right.$$

For matching regions with multiple minimum SSDs, the process is no longer a random selection of images, or of the first or last image piece encountered in a circular search, which allows for some shortcomings to be avoided. However, compared with Kim et al. [38], selecting our matching image according to the local minimum total variation is a reasonable criterion for use in selecting *K* images from the film, rather than simply the *K* optional image slices of the weighted average; we can thus avoid image blurring caused by humans.

The proposed algorithm is thus an image classification processing model using auxiliary classifier generative adversarial networks. It is outlined in detail in Algorithm 1 below.

**Algorithm 1.** CP-ACGAN  Step 1: Reading the image *f* and the area mask *M*;  Step 2: According to the ACGAN model, the structure image of *u* is obtained by image *f*;  Step 3: Determine the set of image pixels on the ∂Ω to be classified on the boundary of *S*;  Step 4: For the structural image *u* and *p* to be patched, each p∈∂Ω is centered from an image slice. According to Equation (13), the confidence item *C(p)* is calculated. According to Equation (14), data item *D(p)* is calculated, while priority *P(p)* is calculated according to Equation (15).  Step 5: Determine the highest priority point *P*, as well as the corresponding image block *W* in the corresponding $\psi_{p}$, and record the location of $\psi_{p}$.  Step 6: According to the optimization model from Equation (16), we determine the optimal matching block $\psi (\hat{p})$ and location information in $\psi_{p}\leftarrow \psi (\hat{p})$, then replace $\psi (\hat{p})$ with $\psi_{p}$ to complete the repair of *p* point’s image slices. Meanwhile, in the *u* of structural components, we have used $\psi (\hat{p})$ images to replace the corresponding images of *p* points corresponding to *u*.  Step 7: Update *M* and $\psi_{p}$; Step 8: Determine whether the mask *M* is empty. If it is empty, the algorithm ends; otherwise, return to step 3.

The article "The Novel Sensor Network Structure for Classification Processing Based on the Machine Learning Method of the ACGAN" was retracted in 2020. Reasons: plagiarism; overlap with other authors' work.

## 4. The Experimental Results and Analysis

To further verify the effectiveness of the proposed algorithm, experiments were carried out on the MNIST [35] dataset, the CIFAR10 [36] dataset and the CIFAR100 [39] dataset. In all experiments, the pooling layer in the CP-ACGAN method utilized the averaging pooling method.

The Monte Carlo method [40] is called a stochastic simulation method, sometimes called a random sampling technique or a statistical testing method. It is a mature simulation method. Based on probability theory and mathematical statistics, the Monte Carlo method uses a computer to perform statistical experiments on random variables and random simulations to solve a numerical solution of the approximate solution of the problem. In order to solve the specific problem of image classification, we first needed to establish a probability model or stochastic process related to the solution, whose parameters are equal to the solution of the problem. We then needed to improve the model according to the characteristics of the model or process, and random simulation. The observation or sampling testing process calculates the statistical characteristics of the relevant parameters, and it gives the approximated value and its accuracy.

According to the size of datasets and the experimental conditions of image classification, we chose the Monte Carlo method for random selection of training and testing samples on the CIFAR10 and CIFAR100 datasets. The MNIST dataset is a very classic dataset in the machine learning field. It is ideal for a single-sample testing procedure. The GPU environment was as follows: (1) operating system: Windows 10; (2) GPU: GTX1050+CUDA9.0+cuDNN; (3) IDE: Pycharm; (4) Framework: Pytorch-GPU; (5) Interpreter: Python 3.6.

The article "The Novel Sensor Network Structure for Classification Processing Based on the Machine Learning Method of the ACGAN" was retracted in 2020. Reasons: plagiarism; overlap with other authors' work.

### 4.1. MNIST Dataset Experiment

The MNIST dataset is a handwriting dataset containing a total of 60,000 training samples and 10,000 testing samples. Each sample corresponds to one digit from zero to nine. Each sample has a two-dimensional image dataset 28 × 28 in size, and is expanded into a 784-dimensional vector. To enhance the comparability of our experimental results, the ACGAN network structure of our experiments is described in Figure 3, while the discriminator network structure of the CP-ACGAN is shown in Figure 6. The number of the training epoch was 1000, with one training sample. In the experiments, the generator and discriminator were optimized using the Adam algorithm [41], and the learning rate was 0.002. The experiment also used the deep learning framework and was implemented under a GPU environment.

For existing image classification problems, the most effective and optimal method at present is the DCNN. Thus, the present paper compares the CP-ACGAN method with the CNN method. Because the CNN method differs from the ACGAN model discriminator only in that the pooling layer is added behind the convolutional layer of the CNN, the network structure of the discriminator is exactly the same as that of the CP-ACGAN method. Therefore, in order to make the experiments more comparable, the meaning, minimum and maximum pooling of the CNN were compared.

Figure 7 presents the effect of different methods on the MNIST training dataset after a single sample has 1000 training epochs. The training accuracy [23,24,26,27] of the ACGAN method fluctuates greatly, although the fluctuation range decreases as the number of training epoch increases. In this paper, the CP-ACGAN method reduced the fluctuation range of training accuracy, and the oscillation range reduced rapidly with an increasing number of training procedures. As can be seen from Figure 7, the CP-ACGAN method achieves better convergence than the ACGAN method, and the number of training epochs can quickly be brought down to the desired value with a little training.

Figure 8 presents a testing accuracy comparison of different methods on the MNIST testing dataset [37,42,43]. Under these conditions, the CP-ACGAN can obtain better testing accuracy than the ACGAN. Comparing the mean value of the CNN with the maximum value of the CNN, the accuracy of the CP-ACGAN method can be observed to be higher than this range in most cases.

Table 1 presents the highest accuracy of the different methods on different datasets (MNIST, CIFAR10 and CIFAR100) after 1000 training epochs.

Moreover, Table 2 shows the average prediction accuracy and variance of the different methods when the network training tends to be stable after testing for 1000 epochs.

The article "The Novel Sensor Network Structure for Classification Processing Based on the Machine Learning Method of the ACGAN" was retracted in 2020. Reasons: plagiarism; overlap with other authors' work.

When Figure 8, Table 1 and Table 2 are combined, it is easy to see that the CP-ACGAN method exhibits smaller variance than the ACGAN method, meaning that it has better training and testing stability. At the same time, the maximum prediction accuracy of the CP-ACGAN is 99.61%, which is higher than the 99.45% achieved by the ACGAN, while the average prediction accuracy of 500 epochs is also higher. Compared with the CNN method, the CP-ACGAN method achieves better maximum prediction accuracy and average prediction accuracy than the mean and maximum pooling CNN. However, compared with the CNN method, the variance of the CP-ACGAN method is greater; that is, the stability is slightly worse. Figure 9 presents the images generated by the ACGAN and CP-ACGAN after the completion of 1000 training epochs.

An interesting phenomenon can be observed from Figure 9: namely, although the CP-ACGAN achieves better classification performance, it is worse than the ACGAN at generating images, which is exactly the same as the conclusion drawn regarding GAN-based semi-supervised learning. This problem seems to be a paradox, but as it is based on common problems with GAN supervised learning and semi-supervised learning, it will also be the focus of future work.

### 4.2. The CIFAR10 Dataset Experiment

The CIFAR10 dataset contains more complex data than the MNIST dataset. Each image is a 32 × 32 color image, with an image size of 3 × 32 × 32. There are ten categories, each containing 5000 training images (that is, a total of 50,000 training images), as well as another 10,000 testing images overall. The network structure of the experiment is exactly the same as that of the MNIST’s experimental structure, except for the fact that the output characteristic number of the final output layer of the generator is three, while the input characteristic of the discriminator is also three.

According to the scale of the CIFAR10 dataset, we randomly selected 1000 training samples (including 10 categories) from 50,000 training images using the Monte Carlo method. For the selected training images, the CNN_mean, CNN_max, ACGAN and CP-ACGAN methods were used for every training procedure. The average classification accuracy of the training phase is shown in Figure 10. Figure 10 presents the effects of various methods on the CIFAR10 training classification accuracy after 1000 training samples.

Moreover, Figure 11 presents a comparison of different methods on the CIFAR10 testing dataset. On the CIFAR10 testing dataset, the CP-ACGAN obtains better testing accuracy than the ACGAN. When the mean value of the CNN is compared with the maximum value of the CNN, the testing accuracy of the CP-ACGAN method meets this range in most cases. The testing accuracy of the ACGAN method is almost entirely outside the scope. In the CIFAR10 testing dataset, the random number generated by the Monte Carlo method [40] and the image classification testing image samples partially deviate, but the difference is not significant. The advantage of the Monte Carlo method is that it can be quickly simulated to generate experimental data. The 1000 testing samples used in Figure 11 were selected according to the Monte Carlo method, and the curve in Figure 11 was selected by the Monte Carlo fitting analysis method. From the probability density function, the random number conforming to the normal distribution was calculated.

The article "The Novel Sensor Network Structure for Classification Processing Based on the Machine Learning Method of the ACGAN" was retracted in 2020. Reasons: plagiarism; overlap with other authors' work.

The highest accuracy rates [44] obtained on the CIFAR10 testing dataset after the completion of various training methods and various testing samples in the testing dataset are shown in Table 3. As an example, Table 3 presents the average prediction accuracy and variance of different methods after 1000 tests.

Through analysis of Figure 11, Table 1 and Table 3, we can see that the ACGAN method achieves good results on MNIST; however, when faced with a complex CIFAR10 dataset, the effect is very poor, and far inferior to that of the CNN method. By contrast, the CP-ACGAN method shows strong adaptability. When facing the complex CIFAR10 dataset, the obtained effect is also much better than the CNN method with the same structure; however, the stability is again deficient.

### 4.3. The CIFAR100 Dataset Experiment

CIFAR100 is a dataset similar to CIFAR10, containing three-channel colorful images. However, CIFAR100 has 100 categories with 500 training pictures for each category; that is, 50,000 training pictures, and 10,000 testing pictures. At this time, the number of training samples per-category is less, so the performance of the testing dataset is also slightly worse. The network structure of all classification methods in the CIFAR100 experiment is exactly the same as that in the CIFAR10 and MNIST experiments.

According to the scale of the CIFAR100 dataset, we randomly selected 1000 training samples (including 100 categories) from 50,000 training images using the Monte Carlo method. For the selected training images, the CNN_mean, CNN_max [45], ACGAN and CP-ACGAN methods were used for the training procedure. The classification accuracy effect of different methods on the CIFAR100 training dataset after training 1000 samples is shown in Figure 12.

Figure 13 presents a comparison of different methods on the CIFAR100 testing dataset. Under these conditions, the CP-ACGAN can obtain better testing accuracy than the ACGAN. Moreover, when comparing the mean value of the CNN with the maximum value of the CNN, the accuracy of the CP-ACGAN method exceeds this range in most cases. The classification accuracy of the ACGAN method is almost entirely outside the scope. Compared with the CIFAR10 testing suite, the comparison results of different methods on the CIFAR100 testing suite are smoother, and the ACGAN method performs better.

The article "The Novel Sensor Network Structure for Classification Processing Based on the Machine Learning Method of the ACGAN" was retracted in 2020. Reasons: plagiarism; overlap with other authors' work.

In the CIFAR100 testing dataset, the random number generated by the Monte Carlo method [40] and the image classification testing image samples partially deviate. The advantage of the Monte Carlo method is that it can be quickly simulated to generate experimental data. The testing samples used in Figure 13 were selected according to the Monte Carlo method, and the curve in Figure 13 was selected by Monte Carlo fitting analysis method.

Table 4 reflects the average predictive accuracy [46,47,48] and variance of various methods when training is conducted over 1000 tests and the network is gradually stabilized.

Analysis of Figure 13, Table 1 and Table 4 demonstrates that the ACGAN is similar to CIFAR10, in that the ACGAN is also less effective at dealing with the complex CIFAR100 dataset compared to the CNN with the same structure. The CP-ACGAN method presented in this paper also shows strong adaptability to the CIFAR100 dataset. Compared with the CNN with the same structure, the testing results are greatly improved, and the stability is also improved.

In summary, the ACGAN and CP-ACGAN achieve good classification effects when faced with a simple MNIST dataset. The ACGAN does not perform as well as the CNN when facing complex high-dimensional data; however, the CP-ACGAN method proposed in this paper also achieves good classification effects for these data. Therefore, the CP-ACGAN method can be seen to have enhanced the adaptability of the network to complex data; moreover, compared with the CNN method with the same structure, the effect is also significantly improved.

### 4.4. The Efficiency Comparison

To further illustrate the effectiveness of the proposed algorithm and evaluate its performance, we analyzed the time complexity [41,44,45,49,50,51,52,53] of the CP-ACGAN and compared it in turn with that of the improved models. In this paper, the time complexity of the proposed algorithm is O(nlogn); the time complexity of the CP-ACGAN is better than the CNN_mean, CNN_max, and ACGAN. With the same number of iterations, the training network of the CP-ACGAN performs better than that of the CNN_mean, CNN_max and ACGAN, while the computational complexity of our method was also greatly reduced relative to the others. In summary, the efficiency of our proposed method is superior to that of both the ACGAN and the CNN model [54].

The article "The Novel Sensor Network Structure for Classification Processing Based on the Machine Learning Method of the ACGAN" was retracted in 2020. Reasons: plagiarism; overlap with other authors' work.

## 5. Conclusions

By analyzing the synthesis principle of the ACGAN’s high-definition image and its discriminator judgment ability, a CP-ACGAN is proposed in this paper. Some changes were made to the original ACGAN in the proposed method, including feature matching, changing the output layer structure of the discriminator, introducing the softmax classifier, reconstructing the loss function of the generator and discriminator by means of semi-supervised learning, and introducing the pooling method into the discriminator. The experimental results have shown that, compared with the original ACGAN method, the CP-ACGAN method achieves better classification performance on the MNIST, CIFAR10 and CIFAR100 datasets, and is also more stable than the others. At the same time, compared with a CNN with the same deep network structure, the classification effect of the proposed method is also better. The advantage of the proposed method is that further study of the diversity of GAN-generated samples will further improve the classification effect, meaning that this method has better scalability than others. An interesting phenomenon that emerged in the experiments is that the CP-ACGAN achieves better classification effects than the ACGAN, but the generated image samples are worse than those of other methods. This coincides with the observed phenomenon in which semi-supervised learning based on GAN also achieves better classification performance, but produces worse images. Moreover, the CP-ACGAN method achieves better classification effects than the CNN method, but exhibits some deficiencies in stability. Therefore, the question of how to further improve the stability of the CP-ACGAN classification method will also be the focus of future research work. In addition, in future work, we need to improve the efficiency and rationality of the CP-ACGAN structure by improving the rationality and feasibility of the structure.

## Figures and Tables

**Figure 1:** The original GAN network structure [9].

**Figure 2:** The ACGAN network structure [16].

**Figure 3:** The generator structure of ACGAN [16].

**Figure 4:** Discriminator structure using an ACGAN.

**Figure 5:** The CP-ACGAN network structure.

**Figure 6:** The discriminator structure of the CP-ACGAN.

**Figure 7:** Classification effect of different methods on the MNIST training dataset.

**Figure 8:** Testing accuracy comparison of different methods on the MNIST testing dataset.

**Figure 9:** Comparison of different methods on the MNIST testing dataset.

**Figure 10:** Average classification accuracy of different methods on the CIFAR10 training dataset.

The article "The Novel Sensor Network Structure for Classification Processing Based on the Machine Learning Method of the ACGAN" was retracted in 2020. Reasons: plagiarism; overlap with other authors' work.

**Figure 11:** Average testing accuracy comparison on the CIFAR10 testing dataset.

**Figure 12:** Average classification accuracy of different methods on the CIFAR100 training dataset.

**Figure 13:** Average testing accuracy comparison on the CIFAR100 testing dataset.

**Table 1:** Best prediction accuracy of different methods on MNIST, CIFAR10, and CIFAR100.

Model	*MNIST*	*CIFAR10*	*CIFAR100*
Mean Pooling *CNN*	0.9951	0.7796	0.4594
Maximum Pooling *CNN*	0.9943	0.7639	0.4283
*ACGAN*	0.9950	0.7306	0.3989
*CP-ACGAN*	0.9962	0.7907	0.4803

**Table 2:** MNIST prediction accuracy mean value, maximum value, minimum value and variance of different methods in 1000 testing epochs.

Model	Mean Value	Maximum Value	Minimum Value	Variance
Mean Pooling *CNN*	0.9949	0.9949	0.9865	6.0 × 10^−9^
Maximum Pooling *CNN*	0.9941	0.9941	0.9865	3.3 × 10^−9^
*ACGAN*	0.9940	0.9945	0.9835	4.1 × 10^−7^
*CP-ACGAN*	0.9956	0.9961	0.9890	1.9 × 10^−7^

**Table 3:** CIFAR10 prediction accuracy. Mean value, maximum value, minimum value and variance of different methods in 1000 tests.

Model	The Number of Testing Samples	Mean Value	Maximum Value	Minimum Value	Variance
Mean Pooling *CNN*	200	0.7654	0.7765	0.5705	3.96 × 10^−6^
	600	0.7665	0.7775	0.5800	3.88 × 10^−6^
	1000	0.7670	0.7795	0.5883	3.79 × 10^−6^
Maximum Pooling *CNN*	200	0.7517	0.7605	0.5800	3.88 × 10^−6^
	600	0.7535	0.7645	0.5890	3.76 × 10^−6^
	1000	0.7550	0.7690	0.5960	3.67 × 10^−6^
*ACGAN*	200	0.7196	0.7305	0.5700	5.88 × 10^−5^
	600	0.7203	0.7335	0.5780	5.76 × 10^−5^
	1000	0.7220	0.7365	0.5890	5.69 × 10^−5^
*CP-ACGAN*	200	0.7682	0.7850	0.6700	3.28 × 10^−5^
	600	0.7699	0.7885	0.6790	3.19 × 10^−5^
	1000	0.7715	0.7905	0.6899	3.14 × 10^−5^

**Table 4:** CIFAR100 prediction accuracy. Mean value, maximum value, minimum value and variance of different methods in 1000 Tests.

Model	The Number of Testing Samples	Mean Value	Maximum Value	Minimum Value	Variance
Mean Pooling *CNN*	200	0.6752	0.7105	0.4000	4.92 × 10^−6^
	600	0.6792	0.7185	0.4500	4.88 × 10^−6^
	1000	0.6810	0.7252	0.4800	4.75 × 10^−6^
Maximum Pooling *CNN*	200	0.6514	0.6750	0.3900	5.25 × 10^−6^
	600	0.6560	0.6790	0.4200	5.18 × 10^−6^
	1000	0.6600	0.6830	0.4500	5.15 × 10^−6^
*ACGAN*	200	0.6188	0.6480	0.4200	4.05 × 10^−5^
	600	0.6212	0.6505	0.4400	4.00 × 10^−5^
	1000	0.6258	0.6595	0.4500	3.96 × 10^−5^
*CP-ACGAN*	200	0.7028	0.7300	0.4700	3.75 × 10^−5^
	600	0.7088	0.7380	0.4900	3.70 × 10^−5^
	1000	0.7122	0.7455	0.5022	3.64 × 10^−5^
